# Hydrodynamic Analysis for the Morphing Median Fins of Tuna during Yaw Motions

**DOI:** 10.1155/2021/6630839

**Published:** 2021-01-02

**Authors:** Xiaohu Li

**Affiliations:** Jiangsu University of Science and Technology, Zhenjiang 212003, China

## Abstract

Tuna can change the area and shape of the median fins, including the first dorsal, second dorsal, and anal fins. The morphing median fins have the ability of adjusting the hydrodynamic forces, thereby affecting the yaw mobility of tuna to a certain extent. In this paper, the hydrodynamic analysis of the median fins under different morphing states is carried out by the numerical method, so as to clarify the influence of the erected median fins on the yaw maneuvers. By comparing the two morphing states of erected and depressed, it can be concluded that the erected median fins can increase their own hydrodynamic forces during the yaw movement. However, the second dorsal and anal fins have limited influence on the yaw maneuverability, and they tend to maintain the stability of tuna. The first dorsal fin has more lift increment in the erection state, which can obviously affect the hydrodynamic performance of tuna. Moreover, as the median fins are erected, the hydrodynamic forces of the tuna's body increase synchronously due to the interaction between the body and the median fins, which is also very beneficial to the yaw motion. This study indicates that tuna can use the morphing median fins to adjust its mobility and stability, which provides a new idea for the design of robotic fish.

## 1. Introduction

According to the difference of thrust-generation mechanisms, fish swimming can be divided into two types: the body and/or caudal fin (BCF) mode and the median and/or paired fin (MPF) mode [1–4]. The basic function of median fins varies greatly between these two modes. In BCF mode, median fins are used to maintain body stability and prevent fish from swaying and rolling [5–7]. However, more and more studies have shown that median fins of certain fish species which are classified as BCF mode also play an important role in maneuvers. The bluegill sunfish may be one of the most widely studied species. Jayne et al. [8], Drucker and Lauder [9], Tytell and Lauder [10], Chadwell et al. [11, 12], Borazjani [13], and Flammang and Lauder [14] discussed the features of the soft dorsal fin of the bluegill sunfish and pointed out that the dorsal fin has the function of accelerating the water around it, increasing hydrodynamic performance and balancing overturning moment; therefore, the stability and maneuverability can be controlled efficiently.

Researches showed that tuna median fins have the similar feature as well. In 2017, Pavlov et al. [15] reported in *science* that the base of both the second dorsal and anal fins of bluefin and yellowfin tunas is the existing specific biohydraulic system which can adjust the area and shape of median fins. Median fins are analogous to hydrofoils producing sideways lift force when the fin plane is at an angle with the fluid flow direction [5]. Morphing median fins have the ability of regulating the hydrodynamic force. Under the control of lymphatic pressure, the dorsal and anal fins erect synchronously from cruising behavior with prevailing rectilinear motion to searching and feeding behavior with frequent changes of motion direction. Inspired by this mechanism, Triantafyllou et al. [16] developed a basic vehicle and employed morphing median fins to control its stability and maneuverability. The result indicated that the biomimetic design of morphing fins for AUV (autonomous underwater vehicle) can enhance maneuverability to a certain degree.

Both tuna and bluegill sunfish can change the area and shape of the median fins. However, their hydrodynamic mechanisms are obviously different. The tuna dorsal fin is an ensemble with nearly uniform rigidity, while the bluegill's is composed of spiny anterior and soft posterior portions, which implement high maneuvering mainly by adjusting the flexible part. Due to the difference in physiological structure, tuna generally change the sweep angles of the dorsal and anal fins, and bluegill can realize oscillation motions of its dorsal fin. Thus, the hydrodynamic theory of sunfish's dorsal fin is not quite suitable for tuna.

As a long-range and high-performance object for inspiring the bionics design [17–19], there are many achievements on hydrodynamic analysis and study of tuna. Wolfgang et al. [20] utilized a 3D computational method to describe the swimming motions of the bluefin tuna and obtained the visualization results of the wake structures and the near-body hydrodynamics. Takagia et al. [21] estimated the dynamic properties of bluefin tuna by CFD (computational fluid dynamics) analysis and pointed out that the glide and upward swimming mode of tuna leads to energy saving during motion. Feilich and Lauder [22] indicated that the shape and stiffness can affect the hydrodynamic performance of a tuna-like tail. Xue et al. [23] carried out a numerical hydrodynamic analysis for a physical prototype imitating the shape of tuna based on the Panel method. Then, Xue et al. [24] discussed the evolvement rule and hydrodynamic effect of fluid field around tuna-like model from starting to cruising. Feng et al. [4] performed a numerical study on the hydrodynamic of tuna swimming and obtain drag coefficient and vortex distribution in C-turn maneuvering. Wang et al. [25] combined experimental and computational methods to study the hydrodynamics of finlets in yellowfin tuna during steady swimming. Macias et al. [26] conduct an assessment of the hydrodynamics of tuna swimming wake flow to identify the main characteristics related to the propulsion performance by CFD methods. However, in all the above studies, the median fins of tuna are either simplified as a fixed structure or removed for various reasons.

Pavlov et al. [15] constructed CAD models of the Pacific bluefin tuna with morphing second dorsal and anal fins and carry out hydrodynamic analysis with a CFD program. By comparing the two morphing states of erected and depressed, the conclusion is drawn that erected fins increase lift force within a range of yaw angles from 1° to 8°, and the increment of lift force results in raised lift-to-drag (*L*/*D*) ratios which may be advantageous at turning maneuvers.

This simulation is innovative, but it can be further improved. Tuna is one of the few fish with two dorsal fins. The CAD models of Pavlov only have the second dorsal and anal fins. In fact, the first dorsal fin can also be regarded as a morphing fin because it can unfold out of groove or fold in the groove [15]. Due to the relatively larger variation of area and shape, the hydrodynamic analysis of the first dorsal fin in different morphing states is also necessary. Moreover, the flow fields around the two dorsal fins will interact with each other and affect the lift and drag forces, since they are very close and both have the ability of changing shapes. In addition, as the median fins are erected, the distribution of the flow field around the body may also change. The interaction between the body and erected median fins is worth discussing because it may have an important influence on tuna's swimming performance.

The main objective of this paper is to clarify the effect of erected median fins, including the first dorsal, second dorsal, and anal fins, on the yaw maneuvers of tuna. This study may provide a new idea for the design of a robotic fish, which is to adjust its yaw maneuverability and stability by means of morphing median fins. This article is organized as follows.  Section 2 introduces the CAD simulation models of tuna, the numerical method of hydrodynamic analysis, and the configuration of simulation parameters.  Section 3 discusses the results of hydrodynamic analysis of the median fins under different morphing states and the interaction between the erected median fins and body. Moreover, the analysis results are compared and validated with other research data. Then, the conclusions are shown in Section 4.

## 2. Materials and Methods

### 2.1. Tuna Model

Taking a real yellowfin tuna as the original mold, the physical prototype is obtained by reverse molding process. The body length (BL) of the tuna prototype is about 1.17 m. With laying mark spots around the body and fins, the tuna prototype is scanned into a point cloud image by using a handheld 3D scanner, as shown in Figure 1. The point cloud image is partially missing because the back of the tuna prototype is black and the laser light cannot be reflected effectively. Moreover, there are scattered pieces in the point clouds, so the image needs to be cleaned and reconstructed. It should be noted that during the reconstruction, the image which is a half body of the yellowfin tuna needs to form a full-body image with symmetry operation. Based on reasonable simplification, the contours of the dorsal, anal, and caudal fins are fitted as sine curves by the least square method, while the contours and sections of the body are polynomial and spline curves. The sine equation of the fitting curves of tuna fins can be expressed as follows:

(1) $$\begin{array}{c} z_{n}=a_{n}\cdot \sin\left(b_{n}x+c_{n}\right). \end{array}$$

The parameters of the fitting curves are shown in Table 1. The second dorsal and anal fins with different morphing states are obtained by rotating their fitting curves about points *O*_*d*_ and *O*_*a*_, respectively. To simplify the CAD model, standard symmetric airfoil profiles (NACA0015) are used for all the fin sections based on the measurement data of chord and thickness [27]. Small deviations from the tuna prototype are made in the body, pectoral and pelvic fins. We believe these simplifications and deviations only have a little influence on overall analysis results because the increment values of the lift and drag of the median fins among different morphing states are more important than the absolute values in hydrodynamic analysis.

During rectilinear cruising, the second dorsal and anal fins of tuna are both depressed, and the first dorsal fin is folded in the groove. In searching and feeding behavior, the second dorsal and anal fins erect synchronously, and the first dorsal fin unfolds out of the groove. The CAD model of tuna with two morphing states is shown in Figure 2. According to the measurement data of Pavlov et al. [15], the sweep angle of the first dorsal fin, second dorsal fin, and anal fin in the erection state is set to 35°, 58°, and 61°, respectively. In the depression state, the sweep angle is set to 0°, 76°, and 79°, respectively.

### 2.2. Numerical Method

As the fish swims, the median fins are subjected to the reaction force of the surrounding fluid. In the previous studies, the median fin is usually simplified as a fixed rigid body, and the dynamic theory of the wing is used to analyze the lift force *F*_*L*_ and drag force *F*_*D*_ [1, 28, 29], as shown in equations (2) and (3). The forces *F*_*L*_ and *F*_*D*_ are easily obtained by measuring the lift coefficient *C*_*L*_ and drag coefficient *C*_*D*_ which are constant under this condition. However, the *C*_*L*_ and *C*_*D*_ of tuna median fins are different with different morphing states due to the change of shape, area, and even rigidity. Thus, it is difficult to derive the hydrodynamic expressions of tuna median fins accurately.

(2) $$\begin{array}{c} F_{L}=\frac{C_{L}\rho S\nu^{2}}{2}, \end{array}$$

(3) $$\begin{array}{c} F_{D}=\frac{C_{D}\rho S\nu^{2}}{2}, \end{array}$$

where *C*_*L*_ and *C*_*D*_ are the lift and drag coefficients, respectively, *ρ* is the density of the fluid, *S* is the projected area of the median fin, and *v* is the swimming velocity of the fish.

In this paper, a numerical method is applied to the hydrodynamic analysis for the tuna and its morphing median fins. The flow field of tuna swimming is simulated with the commercial ISIS-CFD flow solver which adopts the incompressible unsteady Reynolds-averaged Navier-Stokes equations. This solver discretizes the transport equations of tuna swimming by the finite volume method. The velocity field and pressure field of tuna swimming are obtained from the momentum conservation equations and the mass conservation continuity equation. Because of the turbulence phenomenon in fish swimming, additional transport equations are needed to model the turbulence variables which can be discretized and solved in a form similar to the momentum equations [30–33]. This flow solver has several near-wall turbulence models, such as one-equation Spalart-Allmaras model, two-equation *k*-*ε* models and *k*-*ω* models, which can be employed in a variety of fish swimming cases.

Generally, tuna swims in the ocean which is regarded as an incompressible viscous monofluid. If only yaw or turning motions are taken into account, the gravity of tuna in Z direction is assumed to be offset by its buoyancy. Thus, the governing equations of tuna swimming can be simplified as follows:

(4) $$\begin{array}{c} \frac{\partial }{\partial t}\int_{V}\rho dV+\int_{S}\rho \left(U-U_{d}\right)\cdot ndS=0,\\ \frac{\partial }{\partial t}\int_{V}\rho U_{i}dV+\int_{S}\rho U_{i}\left(U-U_{d}\right)\cdot ndS=\int_{S}\left(\tau_{ij}I_{j}-{pI}_{i}\right)\cdot ndS, \end{array}$$

where *V* is the domain of interest, or control volume, bounded by the closed surface *S* moving at the velocity *U*_*d*_ with a unit normal vector *n* directed outward; *ρ* is the density of the control volume; *U* and *p* represent the velocity and pressure fields, respectively; and *τ*_*ij*_ are the components of the viscous stress tensor, whereas *I*_*i*_ and *I*_*j*_ are direction vectors.

The grid of the flow field around the tuna moves synchronously as the tuna swims, so the space conservation law must also be satisfied:

(5) $$\begin{array}{c} \frac{\partial }{\partial t}\int_{V}dV-\int_{S}U_{d}\cdot ndS=0. \end{array}$$

To solve the governing equations in this viscous flow, the no-slip boundary condition is imposed on the tuna models [4]:

(6) $$\begin{array}{c} U^{+}=U=U_{T}+U_{R}, \end{array}$$

where *U* is the velocity vector of the tuna. If the tuna is simplified as a rigid body, the velocity *U* only can be decomposed into two components [34, 35]: the translation velocity *U*_*T*_ and the rotational velocity *U*_*R*_.

For yaw maneuvers, the tuna only swims in the *X*-*Y* plane. The fluid force *F* of the median fin is regarded as the resultant force of two components *F*_*L*_ (or *F*_*y*_) and *F*_*D*_ (or *F*_*x*_), which can be computed by integrating the pressure and viscous forces acting on the fin surface *S* [4, 36].

(7) $$\begin{array}{c} F=\left[\begin{array}{c} F_{x}\\ F_{y} \end{array}\right]=\left[\begin{array}{c} \int_{S}\left(\tau_{1j}I_{j}-{pI}_{1}\right)\cdot ndS\\ \int_{S}\left(\tau_{2j}I_{j}-{pI}_{2}\right)\cdot ndS \end{array}\right], \end{array}$$

where *p* is the pressure vector, *I*_*j*_ is the *j*th component of direction vector, *n* is the unit normal vector, and *τ*_*ij*_ is the viscous stress tensor.

The yaw moment *M*_z_ with respect to the center of mass (COM) can be calculated by the following formula:

(8) $$\begin{array}{c} M_{z}=\int_{S}\left[\;r\times \left(\tau_{1j}I_{j}-{pI}_{1}\right)\cdot n+r\times \left(\tau_{2j}I_{j}-{pI}_{2}\right)\cdot n\;\right]\;dS, \end{array}$$

where *r* is the position vector from the tuna's COM.

The numerical algorithm for the flow field of tuna swimming is described as follows:

1. Define the yaw motion law of the tuna; then the *U*_*R*_ and *U*_*T*_ is imposed
2. Update the tuna position according to the motion law at step *k*
3. Solve the governing equation (4) and the space conservation law (5) with the no-slip boundary condition (6) to obtain the flow field distribution around the tuna model [4]
4. Calculate the hydrodynamic force *F* and yaw moment *M*_*z*_ acting on the median fins according to formulas (7) and (8)
5. Return to (2) at the next step *k* + 1

### 2.3. Parameter Configuration

During yaw or turning maneuvers, the exposed median fins can generate hydrodynamic forces, and the variations of their sweep angles can directly affect the lift and drag, thereby changing mobility. We define the yaw motion as a uniform translation movement superimposed on a rotational movement. The yaw motion law of the tuna can be expressed as follows:

(9) $$\begin{array}{c} U=\left\{\begin{array}{c} U_{Tx}=\nu ,\\ U_{Rz}=\omega \cdot r, \end{array}\right. \end{array}$$

where *v* is the translation velocity in *X* direction, *r* is the position vector from the COM, and *ω* is the yaw angular velocity around *Z* axis.

The computational domain of the flow field is a cuboid with a size of 6 × 4 × 4 m. The tuna model yaws around its COM according to the specified motion law in the domain. The unstructured hexahedral meshes are generated based on HEXPRESS™, as shown in Figure 3. The mesh size of the median fins is less than 3 mm, and that of the tuna body is about 6 mm. The box refinement is applied to refine the cells around the tuna model. When doing computations including viscosity, the boundary layer near the tuna model contains high gradients. To properly capture these high gradients, it is important to have a sufficient number of grid points inside the boundary layer. As no-slip boundary condition is imposed on the tuna model, the suggested *Y*^+^ value is below 1 [33]. According to the Reynolds number and *Y*^+^ value, the first layer thickness of the boundary layer is estimated as 0.003~0.005 mm, and the number of layers is approximately 21~26 with the stretching ratio of 1.3. After automatic optimization by the mesh generator under the above parameter settings, the total cells of the domains are over 1.74 and 1.61 million in the erection and depression states, respectively.

The main simulation configuration is shown in Table 2. The *k*-*ω* SST turbulence model, which combines several desirable elements of original *k*-*ω* and *k*-*ε* models, is the recommended model for all basic hydrodynamic computations in FINE™/Marine [33]. The two major features of this model are a zonal blending of model coefficients and a limitation on the growth of the eddy viscosity in rapidly strained flows. It is suitable for the numerical analysis of tuna swimming. The translation velocity of the tuna model is set as *v* = 10 m/s because the swimming speed of tuna is generally 30~50 km/h. The yaw angular velocity is estimated empirically to be 0.5~1.5 rad/s. Moreover, a simulation case with an angular velocity of 0.01 rad/s is also calculated. Due to the relatively small angular velocity, it can be used to analyze the hydrodynamics of the median fins without high speed yaw maneuvers. The case is called the quasistatic yaw motion in this paper. Other parameters, such as maximum number of iterations, convergence criteria, initial condition, and fluid properties, are set by default or suggested values in FINE™/Marine. These default values satisfy the simulation requirements in most cases, including the hydrodynamic analysis of tuna swimming.

## 3. Results and Discussion

### 3.1. Hydrodynamic Analysis under Quasistatic Yaw Motion

The drag, lift, and *L*/*D* ratio of the anal fin (AF) in the erection and depression states under the quasistatic yaw motion (*ω* = 0.01 rad/s) are obtained by CFD analysis, as shown in Figure 4. It can be seen that both lift and drag forces increase with the increase of the yaw angle (*θ*) in the two morphing states. And both the lift and drag force of the erection state are greater than those of the depression state within a range of yaw angles from 0.3° to 20°. This indicates that the erected anal fin can enhance its hydrodynamic forces. In the early stage of yaw motion, the drag changes slowly, while the lift grows fast. But as the yaw angle increases, the drag rises more and more quickly, while the lift rises slowly. As a result, the *L*/*D* ratio improves rapidly at first and reaches the peak when the yaw angle is about 7°~10°, then decreases gradually. When the yaw angle is below 3°, the *L*/*D* ratio of the erection state is close to that of the depression state. Then, the *L*/*D* ratio of the erection state is relatively higher. At the yaw angle of 8.9°, the maximum value of the *L*/*D* ratio in the erection and depression state is 5.76 and 5.3, respectively. It means that the erected anal fin increases its *L*/*D* ratio by approximately 8.7%.

Figure 5 shows the drag, lift, and *L*/*D* ratio of the two dorsal fins in the two morphing states under the quasistatic yaw motion (*ω* = 0.01 rad/s). On the whole, the hydrodynamic trend of the two dorsal fins is similar to that of the anal fin. The lift and drag of the two dorsal fins increase with the increase of yaw angle as well, and the L/D ratio also grows at first and then reduces gradually. However, their hydrodynamic forces still have some different features. It should be noted that the first dorsal (FD) fin is completely folded into the groove in the depression state, so its lift and drag are regarded as zero. At this moment, only the second dorsal (SD) fin generates hydrodynamic forces. Its *L*/*D* ratio reaches the maximum of 11.7 at the yaw angle of 5.8°. Compared with the anal fin, the second dorsal fin is more active in the depression state.

With the erection of the first dorsal fin, the hydrodynamic performance of the second dorsal fin has changed. Its lift reduces a lot, while the drag decreases a little. Consequently, the *L*/*D* ratio of the second dorsal fin diminishes by about 50% from the peak. In a word, the effect of the second dorsal fin is weakened in the erection state. This is similar to the phenomenon in a marathon that the runners in front can reduce the wind drag of the runners behind under certain conditions. Since the first dorsal fin is not far in front of the second dorsal fin, the flow field of the first dorsal fin can also affect the hydrodynamic performance of the second dorsal fin. When the first dorsal fin is erected, the flow fields of the two dorsal fins are fused together partially. The low-pressure area behind the first dorsal fin extends to the second dorsal fin, reducing the pressure difference between the two sides of the second dorsal fin, which leads to the decrease of its lift and *L*/*D* ratio.

However, the erection of the first dorsal fin makes up for the weakening of the second dorsal fin. The drag and lift of the first dorsal fin are much larger than those of the second dorsal and anal fins. Its *L*/*D* ratio becomes the maximum of 11.2 at the yaw angle of 6.4°, which is also higher than the other two fins. It shows that the erected first dorsal fin plays a dominant role among the three median fins. This result is easy to understand. In the erection state, the area of the second dorsal and anal fin is about 57% and 55.6% of that of the first dorsal fin, respectively. The area increment of the second dorsal and anal fin is about 15% and 15.7%, while that of the first dorsal fin is 100%. The absolute area of the two median fins, as well as the incremental area, is much smaller than that of the first dorsal fin, resulting in less hydrodynamic forces.

Figure 6 is the yaw moment of all the median fins in the erection and depression states under the quasistatic motion (*ω* = 0.01 rad/s). It can be seen that the yaw moments of the second dorsal and anal fins are negative in the two morphing states. This indicates that they have the ability of preventing yaw maneuverability and promoting stability. But the first dorsal fin does have the function of improving mobility. In the state of erection, its yaw moment is positive. Although the hydrodynamic forces of the second dorsal and anal fins are very small, their moments are relatively large due to the longer distance from the COM. Most of the time, the positive moment produced by the first dorsal fin cannot completely offset the reverse moments of the second dorsal and anal fins.

From Figure 2, it can be seen that the first dorsal fin is located in front of the COM, and the second dorsal and anal fins are located behind the COM, which directly results in the opposite yaw moments and different hydrodynamic performance. The above analysis results are in agreement with the opinion of Triantafyllou et al. [16] that median fins can increase the yaw rate only if it is placed in front of the center of yaw motion and behind the aerodynamic center. Compared with the second dorsal and anal fins, the first dorsal fin is the one that can improve yaw mobility.

When the yaw angle *θ* is below 4°, the resultant moment of all the median fins in the erection state is a very small value. It means that within the yaw angles of 0°~4°, the median fins as a whole are nearly in a neutral position, which influence neither maneuverability nor stability. Tuna is good at long-distance cruising and has a relatively rigid body and large turning radius compared with other fish [15]. This may indicate that turning or yaw motions are usually achieved at a relatively small yaw angle. The neutrality of the median fins at small yaw angles may be beneficial for tuna to control swimming behaviors, making it easier to trade-off between maneuverability and stability.

The hydrodynamic analysis of each of the three median fins in the two morphing states has been performed above. More importantly, to what extent can the hydrodynamic force of the median fins affect the swimming performance of tuna. Without considering the pectoral, pelvic, and caudal fins, we define the fin-to-body (*F*/*B*) ratio as the ratio of the sum of the hydrodynamic forces of all three median fins to the hydrodynamic force of tuna's body. As shown in Figure 7, within a range of yaw angles from 0.3° to 20°, the *F*/*B* lift ratio is about 16.9%~25.7% and 29.9%~45.7% in the depression and erection states, respectively. The *F*/*B* drag ratio is about 7.5%~17.1% and 22.1%~38.3%, respectively. It can be seen that due to the involvement of the first dorsal fin, the *F*/*B* ratio increases greatly in the erection state, and the hydrodynamic forces of the three erected median fins have reached such a level that it cannot be ignored. Moreover, when the yaw angle is small, the curve of *F*/*B* lift ratio is at a relatively high position, while that of the *F*/*B* drag ratio is relatively low. It means that the median fins have greater influence on the yaw motion of tuna at the small yaw angles. As discussed above, this may be an optimization of the median fins for swimming control at small inclination yaw motions.

### 3.2. The Body-Fin Interaction

It needs to be noted that the erection of the median fins affects not only themselves but also the hydrodynamics of the tuna's body. As shown in Figure 8, the lift and drag force of the body also increase, when all the median fins are erected. And the maximum value of the *L*/*D* ratio of the body rises from 4.3 to 5.1 at the yaw angle of 9.3°. An increase of 18.6% in the *L*/*D* ratio is very beneficial for tuna in searching and feeding behaviors. Since the tuna's body is exactly the same in the two morphing states, we believe that the body-fin interaction is responsible for the raised *L*/*D* ratio. This is in agreement with the viewpoint of Liu et al. [37]. By comparing the body-median-fin model and the body-only model, they have drawn the conclusion that the body-fin interaction improves thrust in swimming fishes. It is slightly different from this paper. Their conclusion focuses on the influence of the presence or absence of the median fins on the hydrodynamic forces, while we are concerned about the effect of the morphing states of the median fins. After a long period of evolution, tuna has become a complex and sophisticated system. Any change in its morphological structure may cause obvious changes in the overall performance. The morphing states of the median fins have an important influence on the body's hydrodynamic forces, thus further affecting the swimming performance of tuna.

One reliable explanation about the body-fin interaction is that the pressure distribution around the body changes as the median fins is erected.  Figure 9 is the pressure contours of the body in the two morphing states at the yaw angle of 9.5°. The coordinate of the cut plane is *z* = 0.12 m, which is closer to the dorsal fins. When the first dorsal fin is folded into the groove, the pressure field around the body on the cut plane is even. With the erection of the median fins, the pressure of the front edge of the body's upstream surface increases, while the pressure on the downstream surface decreases, thereby enlarging the pressure difference between the two sides of the body. This is the direct cause of the increase in the lift and *L*/*D* ratio. Another phenomenon also can be seen from Figure 9. Compared with the erection state, the flow field around the second dorsal fin appears obvious high-pressure and low-pressure areas in the depression state. This further confirms that the second dorsal fin has less hydrodynamic forces in the erection state.

Figure 10 is the lift and drag increments in the erection state. It can be seen that the lift increments of the second dorsal and anal fins are relatively small. It seems that changes in their own hydrodynamic forces can hardly have a significant impact on tuna's mobility. When the yaw angle is small, the lift increment of the first dorsal fin is the largest, followed by the body. They work together to enhance the swimming performance of the tuna. As the yaw angle increases, the lift increment of the body is even greater, and its drag increment is relatively less than that of the first dorsal fin. Gradually, the body has more efficient hydrodynamic performance. It implies that the body-fin interaction, rather than the median fins themselves, may be one of the important reasons for improving mobility in the erection state.

As shown in Figure 11, from the perspective of moment increment, the first dorsal fin and the body still play an important role in promoting yaw maneuvers. Their moment increments are usually larger than those of the second dorsal and anal fins. As mentioned above, the moments of the second dorsal and anal fins are negative. In the erection state, due to the decrease of hydrodynamic forces of the second dorsal fin, its reverse moment reduces, which is equivalent to an increase in the positive moment. But the anal fin produces more reverse moment, which further inhibits the yaw motion. The sum of their moment increments is very small within the yaw angles of 0°~9°. It indicates that the erection of the second dorsal and anal fins has limited effect on yaw maneuvers when the yaw angle is below 9°.

### 3.3. Hydrodynamic Analysis during Yaw Maneuvers

Different from the quasistatic motion, the yaw maneuvers have a higher angular velocity. With the increase of the yaw speed, the hydrodynamic characteristics of the median fins change in some aspects. As shown in Figure 12, the *L*/*D* ratios of the anal fin rise rapidly to the maximum values when the yaw angles are about 2.5°~5.5° in the two morphing states. Compared with the quasistatic condition, the peak values of *L*/*D* ratio appear earlier. This is in line with the characteristic of tuna's small-inclination axial movement and is more conducive to the quick intervention of the median fins in the yaw maneuvers. When the angular speed is 0.5 rad/s, 1.0 rad/s, and 1.5 rad/s, the corresponding maximum value of the *L*/*D* ratio in the erection state is 7.1, 10.0, and 14.7. And in the depression state, it is 7.6, 13.1, and 17.9, respectively. Obviously, this shows two points. One is that the *L*/*D* ratio increases with the increase of the yaw speed under the same morphing state. The other is that the *L*/*D* ratio of the erection state is smaller than that of the depression state at the same speed. Similar to the anal fin, the *L*/*D* ratio of the second dorsal fin in the erection state is also reduced, and the reduction is more significant. The maximum *L*/*D* ratio of second dorsal fin in the depression state can reach 12.8, 13.9, and 15.4, with the corresponding yaw speed of 0.5 rad/s, 1.0 rad/s, and 1.5 rad/s. But in the erection state, it is reduced to 6.6, 7.7, and 9.8, respectively. Due to the negative effect of the first dorsal fin, its *L*/*D* ratios decrease by about 36~48%. It can be seen that the erection of the anal and second dorsal fins only raises the lifts and drags, not the *L*/*D* ratios. In other words, the drag force increases more than the lift force in the erection state. It is not beneficial to the improvement of hydrodynamic performance.

Moreover, the lift increment of the erected anal fin is a positive value during the yaw maneuvers, while that of the erected second dorsal fin is a negative value. The sum of their lift increments is nearly zero, so the effects on tuna's mobility almost cancel each other out. Similarly, the moment increments also offset each other. From the perspective of lift and moment increment, the erection of these two median fins does not directly improve the tuna's mobility during the yaw maneuvers. This is consistent with the previous conclusion. The median fins of a tuna are analogous to the morphing wing of an aircraft. According to the wing theory, the morphing wing can optimize the flight performance of the aircraft at high and low speeds. The erected wing is mainly used to improve stability at low speed rather than maneuverability. By the same principle, the erection of the second dorsal and anal fins may be more inclined to improve the stability of the tuna rather than its yaw maneuverability.

As shown in Figure 13, the maximum *L*/*D* ratios of the first dorsal fin decrease slightly with the increase of the yaw speed. When the velocity is 0.5 rad/s, 1.0 rad/s, and 1.5 rad/s, the corresponding value is 9.7, 10.2, and 10.7, respectively. The *L*/*D* ratio of the body is usually larger in the erection state than that in the depression state at any given angular velocity. And the maximum values of *L*/*D* ratio increase by about 10~18% in the erection state. No matter which state the body is in, the *L*/*D* ratio curves converge at an intersection point. The yaw angle of the point is 5.9° in the erection state, while it is 7.3° in the depression state. When the yaw angle is less than the point, the *L*/*D* ratios increase with the increase of the yaw speed; otherwise, they decrease with the increase of the angular velocity.

The lift increments of the first dorsal fin and body do not vary much with different yaw speeds when the yaw angles are below 9°. They are much larger than the lift increments of the second dorsal and anal fins, which are enough to affect the swimming performance of tuna. These further confirm that the first dorsal fin and the body-fin interaction are the two main ways to improve the hydrodynamic forces in the erection state.

Tuna has two dorsal fins, and their functions are different due to the different positions. The first dorsal fin is located in front of the COM, and its hydrodynamic forces can provide positive moment for yaw motions, while the second dorsal fin is opposite. This may provide a new bionic idea for the design of robotic fish. Most of the existing robotic fish that mimic the BCF swimming mode have only one fixed dorsal fin. Inspired by this mechanism, we can use two morphing dorsal fins to balance the maneuverability and stability of the robotic fish by adjusting their erection or depression states.

### 3.4. Comparative Verification

A mesh independence study is conducted by using three different sets of grids in the depression state, which have about 1.24 (coarse), 1.61 (medium), and 2.56 (fine) million cells, respectively.  Figure 14 is the *L*/*D* ratio of the body with different grids at the same yaw speed of 0.01 rad/s. It can be seen that the three sets of simulation data are very close to each other. Taking the results of the fine grid as reference, the maximum error of the coarse grid and medium grid is about 2.51% and 2.1% within a range of yaw angles from 0.5° to 20°, respectively, and the mean error is about 0.96% and 0.4%. The accuracy of the medium mesh used in this paper is acceptable and does not affect the correctness of the conclusions above. It shows that these simulations are mesh independent.

To verify the reliability of current results, it is compared with the simulation data of Pavlov et al., as shown in Figure 15. On the whole, the trend of *L*/*D* ratio curves is similar. The *L*/*D* ratios of the second dorsal fin increase quickly when the yaw angle is small and reach the maximum values within a range of yaw angles from 4.5° to 7.5°, then decrease gradually to about 2~3.5. Basically, the trend is also consistent with the test data of the morphing aquatic micro air vehicle [38], which can change sweep the angle of its wing during the flight. This shows that the simulation results of this paper are credible to a certain extent.

Due to the differences of CAD models, the absolute values of *L*/*D* ratios are different between current results and Pavlov's data. The model in this paper is based on a yellowfin tuna and uses NACA0015 airfoil as the cross-section of all the fins, while the model of Pavlov is constructed without some details of a bluefin tuna morphology, including the first dorsal and pelvic fins [15]. As mentioned above, the presence of the first dorsal fin weakens the *L*/*D* ratio of the second dorsal fin, which causes an obvious difference in the erection state. In addition, the simulation in this paper is carried out at the yaw speed of 0.01 rad/s, while the Pavlov's data are obtained under static conditions. This is also one of the reasons for the difference. Under different modeling and computational methods, it is a common phenomenon that there are some discrepancies in the absolute values of simulation results. However, relative values are the focus of this paper. What we care about is the lift and *L*/*D* increments between the erection and depression states. In fact, the increment values of *L*/*D* ratios are close to each other. The *L*/*D* increment of the erected anal fin in this paper is about 8.7%, and Pavlov's result is about 11%. This is also similar to the data of Siddall et al. [38]. And we all came to the same conclusion that the erected median fins could increase their own lifts to a certain extent. This further verifies the simulation results in this paper. But it should also be emphasized that our views do not coincide in some aspects. Pavlov et al. pointed out that the erected second dorsal and anal fins may facilitate turning maneuvers, but the analysis result of this paper shows that only the first dorsal fin can improve maneuverability.

## 4. Conclusion

On the basis of scanning and measuring the physical model of real yellowfin tuna, the CAD simulation models with two morphing states of the median fins are constructed in this paper. The hydrodynamic analyses of the median fins under different morphing states are carried out by numerical method, to clarify the influence of the median fins on the yaw motion of tuna. Through the discussion of the simulation results, the following conclusions can be drawn:

1. The erection of the median fins can improve the hydrodynamic forces. The *L*/*D* ratio of the erected anal fin increased by a maximum of 8.7%. Due to the negative impact of the first dorsal fin, the hydrodynamics of the second dorsal fin is reduced in the erection state. The second dorsal and anal fins are located behind the COM and produce a reverse yaw moment. Their resultant lift and moment change a little between the two morphing states, so the effect on the yaw mobility of tuna is limited
2. Because of the larger area increment of the first dorsal fin, its hydrodynamic increment in the erection state is much larger than that of the second dorsal fin and anal fin. And the first dorsal fin located in front of the COM can generate positive yaw moment, which is beneficial to enhance the yaw performance of tuna. Thus, it is believed that among the three median fins, the erected first dorsal fin plays a leading role in improving yaw mobility
3. In addition to raising their own hydrodynamic forces, the erection of the median fins also affects the hydrodynamics of the body. When all median fins are erected, the distribution of the flow field around the body changes, increasing its lift force and yaw moment. This body-fin interaction also has an important effect on the yaw maneuvers, further improving the hydrodynamic performance of the tuna. This indicates that compared with the second dorsal fin and anal fin, the erected first dorsal fin and body-fin interaction have more significant effects to improve the yaw mobility of tuna

According to the above analysis results, it is reasonable to believe that the second dorsal and anal fins tend to maintain yaw stability of tuna, while the first dorsal fin helps to improve yaw mobility. Based on this bionic principle, the three morphing median fins can be designed for robotic fish to facilitate the control of their yaw maneuverability and stability. In future studies, we will apply this mechanism to AUVs.

## Figures and Tables

**Figure 1:** The physical prototype of a yellowfin tuna. (a) Scanning the physical prototype with a 3D scanner; (b) the point cloud image; (c) the fitting curves of the tuna model.

**Figure 2:** The morphing states of the median fins. (a) All median fins are erected. (b) All median fins are depressed.

**Figure 3:** The unstructured hexahedral meshes of the flow field and tuna model: (a) the volume mesh of the flow field and (b) the surface grid of the tuna model.

**Figure 4:** The drag, lift, and *L*/*D* ratio of the anal fin (AF) in the erection and depression states under the quasi-static yaw motion (*ω* = 0.01 rad/s): (a) the drag of the anal fin; (b) the lift of the anal fin; (c) the *L*/*D* ratio of the anal fin. Note: AF-E (or AF-D) represents the erection (or depression) state of the anal fin.

**Figure 5:** The drag, lift, and *L*/*D* ratio of the first dorsal (FD) and second dorsal (SD) fin in the erection and depression states under the quasi-static yaw motion (*ω* = 0.01 rad/s): (a) the drag of the two dorsal fins; (b) the lift of the two dorsal fins; (c) the *L*/*D* ratio of the two dorsal fins. Note: FD-E represents the erection state of the first dorsal fin; SD-E (or SD-D) represents the erection (or depression) state of the second dorsal fin.

**Figure 6:** The yaw moment of the median fins in the erection and depression states under the quasi-static yaw motion (*ω* = 0.01 rad/s): (a) the respective moment of all the median fins; (b) the resultant moment of all the median fins.

**Figure 7:** The *F*/*B* ratio in the erection and depression states under the quasistatic yaw motion.

**Figure 8:** The drag, lift, and *L*/*D* ratio of the tuna body in the erection and depression states under the quasi-static yaw motion (*ω* = 0.01 rad/s): (a) the drag of the body; (b) the lift of the body; (c) the *L*/*D* ratio of the body. Note: B-E (or B-D) represents the hydrodynamic force of the body (B) when all median fins are erected (or depressed).

**Figure 9:** The pressure contours of the tuna body on the cut plane of *Z* = 0.12 m at a yaw angle of 9.5° in the depression and erection states, respectively: (a) the pressure contour of the body when all the medians are depressed; (b) the pressure contour of the body when all the medians are erected. Note: the white ellipses are the cut sections of the body and second dorsal fin, respectively.

**Figure 10:** The lift and drag increments in the erection state of the body (B), first dorsal (FD), second dorsal (SD), and anal fins (AF) under the quasistatic yaw motion (*ω* = 0.01 rad/s).

**Figure 11:** The moment increments in the erection state of the body (B), first dorsal (FD), second dorsal (SD), and anal fins (AF) under the quasistatic yaw motion (*ω* = 0.01 rad/s).

**Figure 12:** The *L*/*D* ratios and lift increment of the anal and second dorsal fins in the two morphing states with the yaw angular velocity of *ω* = 0.5 rad/s, 1 rad/s, and 1.5 rad/s, respectively: (a) the *L*/*D* ratio of the anal fin; (b) the *L*/*D* ratio of the second dorsal fin; (c) the lift increment of the anal and second dorsal fin.

**Figure 13:** The *L*/*D* ratio and lift increment of the first dorsal fin and the body in the two morphing states with the yaw angular velocity of *ω* = 0.5 rad/s, 1 rad/s, and 1.5 rad/s: (a) the *L*/*D* ratio of the first dorsal fin; (b) the *L*/*D* ratio of the body; (c) the lift increment of the first dorsal fin and the body.

**Figure 14:** The *L*/*D* ratio of the body with different grids (*ω* = 0.01 rad/s; depression state).

**Figure 15:** Comparison of current results with the simulation data of Pavlov: (a) the *L*/*D* ratio of the second dorsal fin; (b) the *L*/*D* ratio of the anal fin.

**Table 1:** The fitting curve parameters.

	*n*	*a*_*n*_	*b*_*n*_	*c*_*n*_	*x*
Second dorsal fin	1	219.4	0.004698	10.51	0.54 ≤ *x* ≤ 0.72
	2	218.5	0.006867	15.16	0.62 ≤ *x* ≤ 0.72
First dorsal fin	3	241.1	0.01156	9.665	0.29 ≤ *x* ≤ 0.36
Anal fin	4	213.3	0.004391	7.40	0.59 ≤ *x* ≤ 0.78
	5	213.8	0.005812	18.74	0.67 ≤ *x* ≤ 0.78
Caudal fin	6	194.4	0.00666	12.25	0.99 ≤ *x* ≤ 1.17
	7	202.8	0.009863	27.17	1.08 ≤ *x* ≤ 1.17

**Table 2:** The simulation parameter configuration.

Parameter		Value
Domain size		6 × 4 × 4 m
Turbulence model		*k*-*ω* SST
Yaw angular velocity		*ω* = 0.01, 0.5, 1.0, 1.5 rad/s
Translation velocity		*v* = 10 m/s
Time step		*∆t* = 5.0*e*^−2^, 1.0*e*^−3^, 5.0*e*^−4^, 3.3*e*^−4^s
Convergence criteria		2 orders
Maximum number of iterations		20
Total number of cells	Erection	1744610
	Depression	1614307

## Data Availability

The data used to support the findings of this study are included within the article.
